# Construction of Correlation Analysis Model of College Students' Sports Performance Based on Convolutional Neural Network

**DOI:** 10.1155/2022/3621316

**Published:** 2022-05-27

**Authors:** Guangtao Jiang

**Affiliations:** Department of Physical Education, Sanquan College of Xinxiang Medical University, Xinxiang 453003, China

## Abstract

This paper proposes a network model recurrent fully connected network (RFC-Net) based on recurrent full convolution and polarization change. RFC-Net enriches the network by reconstructing and fine-tuning the fully convolutional network and adding recurrent convolutions to it. By studying the data mining technology of multidimensional association rules, based on the existing algorithms, this paper improves the shortcomings of the algorithms and realizes an efficient and practical method for data mining based on interdimensional multidimensional association rules. On the basis of mastering the actual student information, the effectiveness of the method is tested, and an employment analysis system based on association rules is established. Aiming at the fact that traditional grade prediction methods ignore the different influences of different behavioral characteristics on grades, and considering that behavioral data in different periods have different influences on student grades, the grade prediction problem is abstracted into a time series classification problem. The mechanism is combined with long short-term memory neural network to construct a performance prediction model based on Attention-BiLSTM. Experiments show that the prediction model proposed in this paper improves the accuracy and effectively improves the prediction quality compared with the logistic regression model with a better prediction effect in the traditional benchmark model and the long short-term memory neural network model without the introduction of the attention mechanism. Research shows that physical performance and academic performance are not contradictory. We must face up to the status of physical exercise in schools; as long as physical exercise is properly arranged, it can inspire students to form a spirit of unity, interaction, positivity, and perseverance in cultural studies.

## 1. Introduction

At the same time, society and schools have a tendency to attach importance to the development of students' intellectual education and despise students' physical education. Students are overburdened with schoolwork, so there is a serious lack of time for rest and exercise. It is an urgent problem to improve society's attention to physical education. In schools, the platform for students to understand physical education and engage in physical exercise is physical education class [1, 2]. In physical education classes, for students, teachers are not only the communicators of students' physical skills but also the communicators of a healthy lifestyle. The evaluation of physical education results directly affects students' attitudes and cognitions to physical education classes and physical education learning. However, the existing physical education performance evaluation has various drawbacks, which can easily cause students' negative emotions and greatly reduce the effect of physical education classes [3, 4]. Only by adopting the method can make students feel the significance of physical education and improve students' enthusiasm, and let students understand and love sports, so as to fundamentally better solve the current situation of students' physical health decline [5, 6].

There is no innovative development and change in the assessment of students' physical education performance in teaching evaluation. In most physical education classes, sports technology is still the main assessment content, and the proficiency in sports technology or the strength of one's own physical fitness is used as the final evaluation standard [7, 8]. Such an evaluation method obviously lags behind the requirements of the current physical education teaching reform. It is difficult to include and reflect on the physical health status of students in the physical education performance evaluation system, thus affecting the overall development of the physical education curriculum and teaching reform [9, 10].

The ideas of facing all students, everyone's participation, and health first should be run through it. However, in the past, the physical education curriculum and teaching evaluation were mainly based on the examination system. Without paying attention to the individual differences of students, ignoring the physical state, learning attitude, effort level, and sports foundation of students, the sports assessment method centered on sports technology alone cannot reflect individual differences, resulting in unfair sports performance evaluation [11].

Association rule mining is one of the important contents of data mining. The data mining of the characteristics and behaviors of groups is an important and complex direction of association rule mining. For example, the association tendency between students' individual natural information and their employment behavior in the student employment system belongs to this kind of situation. However, many common data mining tools at present, based on the consideration of more general mining needs, do not provide sufficient support for the above mining needs. In view of the traditional performance prediction research, this paper only considers the use of historical performance to predict target performance, or only uses a single type of behavioral data to predict target performance, and does not consider the different degrees of influence of different behavioral characteristics on grades. The attention mechanism is introduced to build a performance prediction model, and it is compared with benchmark models such as support vector machine and logistic regression through experiments. There is a significant positive correlation between sports performance and academic performance, indicating that students with high sports performance are also high in academic performance; college students' self-efficacy has a significant positive correlation with sports performance and academic performance.

## 2. Related Work

Relevant scholars proposed to use the parameter reduction feature architecture of a fully convolutional neural network to alleviate this problem [12]. The network architecture is divided into an encoding phase and a decoding phase. The encoding phase uses vertical convolutional layers, horizontal convolutional layers, and fully connected layers. The decoding stage uses four layers of deconvolution horizontal layers and two layers of deconvolution vertical layers [13]. The final experiment proves that increasing the feature similarities and differences between channels effectively improves the performance of the model [14].

Relevant scholars have optimized the LeNet network structure and proposed a deeper and wider AlexNet network structure than LeNet [15]. This network structure uses the dropout layer for the first time to reduce the occurrence of model overfitting, in order to strengthen the network as a whole.

The researchers made further improvements on the basis of the ResNet network structure and proposed the DenseNet network structure [16]. In the DenseNet network structure, a connection relationship is established between each different network layer. This structure can reduce the occurrence of the common gradient vanishing problem during training. In addition, in order to reduce the amount of network parameters and model computation of the network model, the DenseNet network adds a 1 × 1 convolutional layer between the bottleneck layer and each module [17].

The method of measuring students' sports performance only relying on movement technique and physical quality assessment will hinder the development of students' cognition, self-confidence, and interest. The evaluation of college students' sports performance should be adjusted accordingly to meet the requirements of the “new curriculum reform”. It also proposes that the evaluation should reflect the student's dominant position [18, 19].

The researchers pointed out that physical education has undergone great changes mainly around the setting of physical education courses and teaching methods, while the physical assessment has not changed [20]. The degree of mastery is used as the evaluation standard for students' assessment performance. This method can easily reduce the enthusiasm of students to study physical education. In the long run, it will seriously affect the reform of physical education teaching [21].

Relevant scholars pointed out that the differences in students' physical state, learning attitude, effort level, and sports foundation are the objective reflection of students' individual differences in learning results [22]. It is recommended to give the right of evaluation to students, taking into account the individual differences of students. Scholars have also proposed that the factors of individual differences of students should be fully considered in the evaluation of sports performance [23]. If the individual differences among students are ignored, it will not only be detrimental to the development of students and the improvement of the overall educational level but also run counter to the ultimate goal of physical education.

Scholars pointed out that in the process of students learning sports techniques and physical exercises in physical education, there is an objective effect of developing physical fitness and sports quality, and good physical fitness and sports quality are also the basis for students to master sports technology well [24]. Therefore, in physical education courses, whether it is to better master sports techniques or to effectively improve students' physical health, physical education teaching needs to pay great attention to the development of students' physical fitness and sports quality. Middle school students are in the stage of puberty development, which is also an important stage for improving their physical quality.

Students' physical fitness is greatly affected by genetic factors and daily life habits, and individual differences are large. A large number of works of literature related to physical fitness are more about the physical fitness of various sports or athletes, and most of the research on the physical fitness of middle school students is about the factors and countermeasures for the continuous decline of students' physical fitness, and this is about the development of students' physical fitness and physical health. The problem has attracted widespread attention from all walks of life in the society. Good physical fitness and athletic quality are also the basis for students to master sports techniques well [25]. Therefore, in physical education courses, whether it is to better master sports techniques or to effectively improve students' physical health, physical education teaching needs to pay great attention to the development of students' physical fitness and sports quality.

## 3. Methods

### 3.1. Convolutional Neural Network Model

The convolution kernel in the convolutional layer first learns the feature map of the previous layer and then uses the activation function to filter. Each convolutional layer can be represented by the following formula:

(1) $$\begin{array}{c} x_{q}=\int \prod_{i=0}^{I-1}\prod_{j=0}^{M_{i}}\left(k_{ji,q}•x_{j,q-1}+b_{i,q}\right), \end{array}$$

where *x*_*q*_ is the feature map of the *q*th layer. The downsampling layer achieves the effect of increasing the receptive field and reducing the number of features by reducing the resolution of the feature map and outputs the feature map by the following formula:

(2) $$\begin{array}{c} x_{q}=\prod_{i=0}^{I-1}\int \beta_{i,q}\text{downsample}\left(x_{i,q-1}\right)-b_{i,q}, \end{array}$$

where *β* is the downsampling weight, and downsample( ) is the downsampling function. By dividing the feature map into multiple nonoverlapping *d×d* blocks, and then averaging or maximizing the features in each block, the feature maps are reduced by a factor of *d*.

After flattening the two-bit feature map into a one-dimensional feature map, it is used as the input of the fully connected layer.

(3) $$\begin{array}{c} x_{q}=\int \left(w_{q-1}x_{q+1}-b_{q-1}\right), \end{array}$$

where *w*_*q*_ is the weight coefficient and *b*_*q*_ is the bias term.

Shallow layers in convolutional neural networks can extract low-level features such as edges, while deep layers can further extract corners, textures, and complex object-specific features based on the low-level feature information extracted by shallow layers. Usually, the convolutional layer is a max-pooling layer, which reduces the size of the feature map by dividing the feature map into blocks and replacing the entire block with its maximum value.

### 3.2. Fully Convolutional Networks

FCN uses and extends existing sports performance classification models and then fine-tunes the parameters of the convolutional layers with the input of the whole image and the gold standard [15, 26, 27].

The convolutional layers in FCN are translation invariant; that is, the operations of the convolutional layers are only associated with low-level feature maps in the perceptual region [28, 29].

Write a data vector in *x*_*ij*_ for the *(i*, *j)* position in a particular layer and *y*_*ij*_ for the next layer, these functions compute the output *y*_*ij*_.

(4) $$\begin{array}{c} y_{ij}=f_{ks}\left[x_{si-\delta_{i},sj+\delta_{j}}\right]\delta_{i},\;\delta_{j}⟶\left(0,k\right), \end{array}$$

where *k* is called the kernel size, *s* is the stride, and *f*_*ks*_*()* determines the layer type.

### 3.3. Circular Convolution

The input of the recurrent convolutional network is a sequence of length *T*, where *x*_*T*_ represents a vector, the function *h*_*t*_ is used internally, and the output is also a sequence [19]. For each input *x*_*t*_ of the sequence, the same *θ* is used for calculation, and a vector *h*_*t*_ is output.

The operations of a recurrent convolutional layer are performed for discrete time steps expressed in terms of a recurrent convolutional network. For a unit *(i*, *j)* located on the k-th feature map in a recurrent convolutional layer, its net output *M*_*ijk*_*(t)* at time step *t* is given by

(5) $$\begin{array}{c} M_{ijk}\left(t\right)=W_{k,p}^{-1}x_{i,j}\left(t+1\right)-W_{k,q}^{-1}y_{i,j}\left(t-1\right)-b_{k}, \end{array}$$

where *y(t)* and *x(t-1)* represent feedforward and loop inputs, respectively, which are vectorized patches centered on the feature maps *(i*, *j)* in the previous and current layers; *W*_*kq*_ and *W*_*kp*_, respectively, represent the normalized feedforward weights and round-robin weights of the k-th feature map, where *b*_*k*_ is the bias. The first term in the above equation is used for circular convolution, and the second term is used for standard convolution. The output of the recurrent convolutional layer is fed to the standard RELU activation function *f*, denoted as

(6) $$\begin{array}{c} F\left(x,w\right)=f\left[M_{ijk}\left(t\right)\right]=\text{Max}\left[\begin{array}{ccc} -1 & M_{ijk}\left(t\right) & 1 \end{array}\right], \end{array}$$

*F(x*, *w)* represents the output of the recurrent convolutional network, which is used for the convolutional layers in the convolutional encoding and decoding units, respectively.

### 3.4. Recurrent Fully Convolutional Neural Network Model Structure

The training and testing process is shown in Figure 1. The RFC-Net network framework is shown in Figure 2. The design of RB in our method is inspired by recurrent convolutional neural networks [25, 30, 31]. The use of data augmentation and polarization changes alleviates the problem of easy overfitting and low accuracy of the model due to the small size of the dataset.

This study adds a batch normalization (BN) between the convolutional layer and the activation function to normalize the sports score blocks after each batch of training.

### 3.5. Recurrent Block Network Structure

The design of the recurrent module in this method is inspired by the recurrent convolutional network, which makes the network richer by incorporating the recurrent module into each convolutional layer [32–34].

Figure 3 shows different variants of the standard convolutional unit and the recurrent convolutional unit. In the figure, *t* = 2 (0∼2) refers to the circular convolution operation. For the *(i*, *j)* unit located on the k-th feature map in the RCL, its net output at time step *t* is given by

(7) $$\begin{array}{c} z_{k,i,j}\left(t\right)=\text{Sum}\left[W_{k,r}r_{k,i,j}\left(-t\right),W_{k,x}x_{k,i,j}\left(t-2\right)\right]-b_{k}. \end{array}$$

### 3.6. Multidimensional Association Rule Mining Based on Apriori without Candidates

Many variants of the Apriori algorithm have been proposed to improve the efficiency of the original algorithm. One of them is to not generate candidate mining [34, 35].

When mining multidimensional association rules, if it is only based on the original Apriori algorithm, it will also bring the above problem: a large number of candidate frequent predicate sets are generated. Therefore, when describing the interdimensional association rule mining, this paper adopts the improved Apriori algorithm, which does not generate candidate frequent predicate sets.

If the frequent predicate sets all satisfy the minimum support degree and then use the minimum confidence degree judgment, the multidimensional association rules can be easily obtained.

The nonfrequent predicates are immediately discarded during processing and are not stored in the candidate frequent predicate set. Thus, additional overhead is avoided, and efficiency is effectively improved.

This paper expects to discover the cross-relationship between college students' information through multidimensional association rule mining based on Apriori that does not generate candidates.

## 4. Results and Analysis

### 4.1. Model Training Parameter Settings

Considering that some behavioral feature data are relatively sparse, an adaptive model optimization algorithm needs to be selected, and the Adam optimization algorithm has a better convergence effect on the model and can correct the model. Problems such as slow convergence speed during training are also widely used, so the Adam optimizer is selected during model training.

Since the problem of grade prediction is abstracted into a time series classification problem in this study, the commonly used loss function is cross-entropy when dealing with classification problems. Therefore, the binary_crossentropy loss function of binary_crossentropy is determined to be used during model training.

The problem of overfitting is often encountered when training neural networks, and the dropout algorithm can effectively prevent overfitting. When training the model, in each batch of training, the values of some neurons will no longer work under the probability of the set size, thereby enhancing the generalization ability of the model and achieving the effect of regularization to a certain extent. Therefore, the dropout strategy is selected during training to prevent overfitting.

In the experiment of this paper, the values of each parameter during the model training process are continuously tested and adjusted on the training set, and three kinds of experiments are carried out for different parameter adjustments. Although Adam is an adaptive optimizer that can adaptively adjust the learning rate, it is not adaptive in the true sense but corrects the gradient from a statistical point of view. The value of the initial learning rate set will still converge with the model. It can be seen from Figure 4 that when the learning rate is set to 4e-7, the training set loss function takes the lowest value under the same number of iterations, and when the number of iterations is about 90, the loss function drops to the lowest.

It can be seen from Figure 5 that, with continuous iterative training, the change of F1 tends to fluctuate, and when the dropout is around 0.04, the effect is better than other values. We choose the learning rate as 4e-7 and dropout as 0.04. It can be seen from Figure 6 that if the batch value is too large or too small, the results of the F1 value are relatively close. When the batch value is in the middle, the F1 value is relatively increased, so the batch size is selected as 20.

### 4.2. Comparison with Traditional Classification Prediction Methods

We combine the attention mechanism and BiLSTM's performance prediction model constructed in this paper with five traditional methods such as support vector machine (SVM), logistic regression (LR), k-nearest neighbor (KNN), random forest (RF), and decision tree (DT). The benchmark classification prediction model and the BiLSTM model without the attention mechanism were compared, and the weighted average grades at the end of the semester were predicted to verify the effectiveness of the prediction method proposed in this paper. The experimental results of the seven models are shown in Table 1.

From the experimental results in Table 1, it can be seen that the classification prediction model based on the combination of attention mechanism and long short-term memory neural network proposed in this paper is better than the other five traditional prediction methods in predicting final grades based on student behavior data. A good prediction effect has been achieved, which is improved compared to the best traditional prediction method logistic regression and BiLSTM without an attention mechanism. In addition, there are also significant improvements in the three indicators of precision, recall, and F1 value.

On the one hand, the traditional classification prediction method takes each behavioral feature directly as the classification feature input model for learning and training and treats the influence of each behavioral feature on the final grade equally. On the other hand, the whole semester's data of each behavioral characteristic are considered as a whole, and it is not considered that the influence of behavioral characteristics of different periods on grades is also different.

The performance prediction method proposed in this paper introduces the attention mechanism into the long short-term memory neural network BiLSTM. First, the BiLSTM network with a long short-term memory unit can store the previous time series information for a long time, organize the behavior characteristics of the whole semester by month, and extract the time series information. The behavior characteristics of different periods have different degrees of influence on grades. The closer the test period is, the greater the impact of behavioral characteristics on performance. Then, the attention mechanism is introduced to apply the behavioral features of different dimensions to determine which behavioral features play a key role in performance prediction. By considering the time step and feature dimension, the combined use of the attention mechanism and the BiLSTM neural network greatly improves the prediction ability of the model, and the accuracy of the performance prediction is relatively more accurate. The experiment also verifies the effectiveness of the proposed model.

### 4.3. Visualization of Attention Results

In order to more intuitively analyze the different degrees of influence of different behavioral characteristics on grades, this paper visualizes the attention scores of different behavioral characteristics, and the results of attention visualization are shown in Figure 7. The figure shows the attention weights corresponding to different behavioral feature indicators.

As can be seen from Figure 7, among the different behavioral characteristics, the attention weights of the three behavioral characteristics of regular meals, monthly Internet fee, and the number of visits to the library are relatively large, while other behaviors such as monthly consumption amount and consumption frequency are relatively large. The attention weight value of the feature is relatively small, indicating that after adding the attention layer, the attention mechanism has indeed “captured” key features, and the behavioral features with a large degree of influence on the performance are assigned a larger attention weight, and the degree of influence on the performance is low. The behavioral features of the model are assigned smaller attention weights, and the behavioral features with different degrees of influence on the performance are treated differently, which can effectively improve the prediction accuracy of the model.

### 4.4. Correlation Analysis between College Students' Sports Performance and Self-Efficacy

As shown in Table 2, the *P* values of the significant probability values are all 0.000 and less than 0.01. Therefore, the results of the *t*-test show that the difference in sports performance of college students with different self-efficacy reaches a significant level.

The correlation coefficient size and significance test results show that the correlation coefficient between self-efficacy and sports performance is *r* = 0.516, and the significance probability value is 0.000 and less than 0.01. It can be concluded that there is a close correlation between college students' self-efficacy and sports performance, and there is a significant positive correlation. According to the one-way analysis of variance of sports performance with different self-efficacy, a linear graph was made to test the changes in different self-efficacy and sports performance. The correlation between different self-efficacy and sports performance is shown in Figure 8.

### 4.5. Correlation Analysis of College Students' Sports Performance and Academic Performance

Participating in physical exercise has a positive effect on the formation of good psychological qualities of college students. The reasons are as follows.

First, as long as the time and intensity of physical exercise are properly arranged, it can support and promote the learning of cultural lessons. Because participating in physical exercise can promote the growth and development of the brain and improve the function of the brain, people who often participate in exercise have a faster response speed of the cerebral nerves and a stronger comprehensive analysis ability of the cerebral cortex.

Second, the reasonable arrangement of physical exercise can cultivate students' strong will, promote students to form good-will qualities such as decisiveness, consciousness, tenacity, and self-control, and finally lay a solid ideological foundation for improving the learning of cultural courses.

Third, reasonable arrangements to participate in collective physical exercise can enable students to create a collective learning environment, which can cultivate students' ideological qualities of caring for the collective, loving the collective, helping each other, and solidarity.

Under the exam-oriented education system, what schools and teachers want is the admission rate, and parents blindly follow suit, so that most teachers only pay attention to the students' test scores in cultural courses, while students' physical quality has been neglected. According to the purpose and requirements of the physical education entrance examination, schools are led by sports backbones to organize students every day outside of class to provide necessary guidance and supervision and plan and reasonably arrange students to participate in healthy physical activities, so that students have ample energy after exercise. We conduct the following analysis on whether there is a contradiction between sports performance and academic performance. As shown in Table 3, the *P* values of the significant probability values are all 0.000, which is less than 0.01. Therefore, the *t*-test results show that the difference in academic performance of college students with different sports scores reaches a significant level.

The correlation coefficient size and significance test results show that the correlation coefficient between sports performance and academic performance is *r* = 0.479, and the significant probability value is 0.000, which is less than 0.01. It can be concluded that there is a close relationship between college students' physical performance and academic performance, and there is a significant positive correlation. According to the one-way analysis of variance of different sports performance and academic performance, a linear graph was made to test the change in academic performance of different sports performance. The correlation diagram between different sports performance and academic performance is shown in Figure 9.

### 4.6. Correlation Analysis of College Students' Sports Performance with Self-Efficacy and Academic Performance

The correlation coefficient size and significance test results show that the correlation coefficient between self-efficacy and sports performance and academic performance is *r* = 0.603, and the significant probability value is 0.000 and less than 0.01. It can be concluded that the self-efficacy of college students is related to sports performance, and there is a significant positive correlation. It shows that students with high self-efficacy have high sports performance and academic performance.  Figure 10 shows the correlation distribution of college students' sports performance with self-efficacy and academic performance.

The level of self-efficacy is an important factor affecting sports performance and academic performance. Therefore, school leaders, physical education teachers, and parents need to fundamentally understand students' sports habits and learning efficiency and formulate exercise plans, study plans, and guidance in a targeted manner, so that students can have the courage and determination to overcome difficulties.

## 5. Conclusion

This paper introduces a recurrent convolutional network, which increases the network depth while keeping the number of tunable parameters constant through weight sharing. The problem of student grade prediction is abstracted as a time series classification problem, and the weighted average grade of students at the end of the term is predicted based on student behavior data. Considering that students' behavior characteristics in different periods have different effects on students' academic performance, different behavior characteristics have different effects on grades. On this basis, combined with the attention mechanism, a grade prediction model is constructed to predict grades, and compared with other benchmark classification prediction models, it is verified that the prediction model proposed in this paper has better accuracy in predicting grades. Research shows that self-efficacy promotes students' willingness to participate in physical exercise, and the level of students' self-efficacy is an important factor affecting sports performance. Therefore, school leaders, physical education teachers, and parents need to fundamentally understand students' physical behavior habits, formulate exercise plans in a targeted manner, and provide guidance, so as to eliminate the adverse factors that restrict students' participation in physical exercise as much as possible, so that students can continuously strengthen students' sports self-efficacy, and promote students to develop the good habit of consciously participating in physical exercise, thereby improving students' sports performance and laying a solid and good foundation for lifelong sports.

## Figures and Tables

**Figure 1:** Training and testing process.

**Figure 2:** Recurrent fully convolutional neural network architecture.

**Figure 3:** Different variants of the standard convolutional unit and recurrent convolutional unit.

**Figure 4:** Function loss convergence diagram.

**Figure 5:** Dropout probability influence diagram.

**Figure 6:** Batch size influence diagram.

**Figure 7:** The effect of various behavioral characteristics on performance.

**Figure 8:** Correlation between different self-efficacy and sports performance.

**Figure 9:** Correlation diagram between different sports performance and academic performance.

**Figure 10:** The correlation distribution of college students' sports performance with self-efficacy and academic performance.

**Table 1:** Comparison of experimental results of different models.

Model	Random forest	Decision tree	KNN	SVM	Logistic regression	BiLSTM	Model of this paper
F1-value	0.64	0.61	0.65	0.67	0.72	0.83	0.89
Precision	0.60	0.64	0.68	0.72	0.73	0.82	0.91
Accuracy	0.72	0.71	0.74	0.68	0.82	0.87	0.92
Recall	0.61	0.66	0.63	0.72	0.74	0.86	0.95

**Table 2:** *T*-test of college students' sports performance with different self-efficacy.

	Excellent	Good	Middle	Poor
Df	401	102	23	2
Standard deviation	6.18	7.65	8.31	2.94
Average	52.21	36.89	28.77	24.12
t	131.22	36.51	16.47	11.63
Sig.	0.000	0.000	0	0.000

**Table 3:** *T*-test of college students' different sports performance and academic performance.

	Excellent	Good	Middle	Poor
Df	301	163	92	44
Standard deviation	42.21	36.86	38.62	41.04
Average	209.45	197.62	186.34	181.11
T	72.01	65.43	91.92	33.94
Sig.	0.000	0	0.000	0.000

## Data Availability

The data used to support the findings of this study are available from the corresponding author upon request.
